# Experimental Study on Hydraulic Pulsation Features of Intelligent Variable Valve System for Auto Energy Saving

This article has been retracted.

**DOI:** 10.1155/2022/5679520

**Published:** 2022-05-18

**Authors:** Yuliang Xu, Jiadui Chen, Zhenghong Liu

**Affiliations:** ^1^School of Mechanical Engineering, Guiyang University, Guiyang 550005, China; ^2^Key Laboratory of Advanced Manufacturing Technology and Ministry of Education, Guizhou University, Guiyang 550025, China

## Abstract

The electrohydraulic valve system can realize continuous variable valve timing and lift using the flexibility of liquid. However, the existing electrohydraulic valve systems usually rely on a high-speed solenoid valve to control the on and off states of the hydraulic circuit, which pushes up the system cost. This paper introduces a continuous hydraulic variable valve timing and lift system with adjustable volume (CVVTL). Unlike the other electrohydraulic valve systems, the CVVTL does not need a high-frequency servo valve to control each valve but adjusts the valve timing and lift by controlling the system volume. However, the maximum operating speed of hydraulic variable valve systems is limited by the inherent pressure fluctuation. To relax the limit, the authors further studied the pressure fluctuation features of the CVVTL system under various conditions and summarized the harms of the fluctuation. After identifying the causes of pressure fluctuation of the CVVTL system, the authors came up with systematic countermeasures to system pressure fluctuation.

## 1. Introduction

Under the premise of ensuring the automobile power performance, improving the engine work efficiency is an effective means to reduce energy consumption and improve the greenhouse effect. The automotive industry applies several technological solutions to improve the engine work efficiency, such as direct fuel injection, engine downsizing, exhaust gas recirculation (EGR), and variable valve trains (VVT) [1–5]. Among them, the VVT can greatly boost the engine performance by adjusting the timing, lift, and duration of the valve according to the engine working conditions. The variable valve actuation can be achieved using mechanical, electromagnetic, and electrohydraulic valve mechanisms [6–11].

Now, many mechanical valve mechanisms are being used in engines, namely, Honda's Variable Valve Timing and Lift Electronic Control (VTEC), Mitsubishi Innovative Valve timing Electronic Control system (MIVEC), Toyota's Variable Valve Timing with intelligence (VVT-i), and Porsche's VarioCam [12, 13]. Nevertheless, the discontinuous change of valve timing offered by the above mechanical valve mechanisms does not support continuous adjustment of valve timing. For example, in VTEC technology, there are only two or three types of distribution cam profiles, which can only meet the ideal distribution requirements of two or three speed conditions of the engine. It is impossible for an engine with such a mechanical valve mechanism to gain reasonable gas distribution under every working condition.

Electrohydraulic and electromagnetic valve mechanisms can achieve continuous valve timing, lift, and duration at all operating speeds and loads. But the electromagnetic valve systems face several disadvantages: large impact of valve seating, huge size of the electromagnet, serious emission of heat, frequent electromagnetic responses, high energy consumption, as well as complex and expensive system [14–17]. For electrohydraulic valve systems, a high-frequency servo valve is often needed to control the value, such as Fiat's Multiair Valve-Lift System [18] and Lotus's electrohydraulic fully variable valve train (EHFVVT) [19, 20].

To solve the defects of the existing VVT technologies, this paper proposes a continuous hydraulic variable valve timing and lift system with adjustable volume (CVVTL). In the system, the advance angle, retard angle, and duration angle of the valve are adjusted continuously by controlling the time that the oil flows into and out from the valve cylinder. The valve lift is adjusted continuously by controlling the liquid volume flowing into the valve cylinder. The CVVTL system eliminates the need for a high-frequency servo valve, which is required by other electrohydraulic valve systems to control each valve. Hence, the system can work at a higher engine speed than the other electrohydraulic valve systems. However, it was found that the oil pressure of the CVVTL system fluctuates during the high-speed operation, which limits the maximum operating speed of the system. Therefore, the authors further examined the phenomenon, causes, harms, and countermeasures of pressure fluctuation in the CVVTL system. Except Xie et al. [21], virtually no scholar has reported the pressure fluctuations of hydraulic variable valve systems.

## 2. Structure and Working Principle of the CVVTL

### 2.1. Structure of the CVVTL

As shown in Figure 1, the CVVTL is composed of a cam, a cam oil cylinder, a valve oil cylinder, a valve assembly, a phase regulator, a lift regulator, a seating buffer, an oil supply system, etc. Among them, the phase regulator and lift regulator each consists of an oil cylinder, a piston, a spring, a gag lever post, and an adjustment device. The oil supply system involves an oil tank, an oil pump, a check valve, a relief valve, and a pipeline.

### 2.2. Working Principle of the CVVTL

The working principle of CVVTL is as follows [22].

#### 2.2.1. Valve Timing Adjustment

Under the effect of the spring, the phase regulator piston lies at the very front of the phase regulator cylinder, while the cam works in the base circle segment for the gag lever post of the phase regulator at any position in the adjustment range. To adjust the valve timing, it is only necessary to change the position of the gag lever post.

When the cam lift is coming, the cam cylinder begins to pump oil. Since the phase regulator spring has a smaller pretightening force than the valve spring, the oil pumped from the cam cylinder would firstly enter the phase regulator cylinder, until the regulator piston is stopped by the gag lever post. At this stage, the valve keeps still. Therefore, the valve is opened after the adjustment of the gag lever post equals zero, that is, the valve advance angle is decreased. As the cam continues rotating, the oil pressure gradually increases in the system. Once the valve cylinder can overcome the pretightening force of the valve spring, the valve is opened, and the valve opening is gradually increased until the end of cam lift.

The above working process is reversed when the cam works in its fall cure. Since the valve spring has a greater force than the phase regulator spring, the oil of the valve cylinder would firstly return to the cam cylinder, until the valve is seated. After that, the cam continues rotating, and the phase regulator spring drives the oil in the phase regulator to return to the cam cylinder, until the cam returns to the base circle segment. Therefore, the valve is closed before the adjustment of the gag lever post equals zero, that is, the valve retard angle is decreased.

Through the above procedure, the system continuously adjusts the advance angle, retard angle, and duration angle of the valve by controlling the time that the oil flows into and out of the valve cylinder.

#### 2.2.2. Valve Lift Adjustment

Under the effect of the spring, the lift regulator piston lies at the very front of the lift regulator cylinder, while the cam works in the base circle segment for the gag lever post of the lift regulator at any position in the adjustment range. To adjust the valve lift, it is only necessary to change the position of the gag lever post.

When cam works in its lift, and the system oil pressure is large enough to overcome the pretightening force of the valve spring, i.e., to open the valve, the lift regulator piston will enter the idle state, for the lift regulator spring has a larger pretightening force than that of the valve spring. In this case, the oil pumped from the cam cylinder will only flow into the valve cylinder to open the valve. Once the system pressure is large enough to overcome the pretightening force of the lift regulator spring, the oil pressure will move the lift regulator piston, and the oil will start to flow into the lift regulator oil cylinder, until the piston is stopped by the gag lever post of the lift regulator. Therefore, the liquid volume entering the valve cylinder will decrease and so will the valve lift.

The above working process is reversed when the cam works in its fall cure. Since the lift regulator works in the opening of the valve, the lift adjustment has no impact on valve timing. It is apparent that the system can continuously adjust the valve lift by controlling the liquid volume entering the valve cylinder and lift regulator. The volume is controlled by properly adjusting the position of the gag lever post of the lift regulator.

Table 1 shows the optimal intake valve opening angle (IVO), intake valve closing angle (IVC), and valve lift parameters of an in-line four-cylinder gasoline engine at different engine speeds. It can be seen that the optimal parameters vary at different engine speeds.

For the CVVTL, the simultaneous adjustment of the valve timing and lift can be achieved, as the system adjusts the phase regulator piston and lift regulator piston to their reasonable positions, according to the working conditions of the engine. Therefore, the CVVTL will be more intelligent because it can meet the gas distribution requirements of the engine in more conditions.

### 2.3. CVVTL Prototype

This paper develops a four-cylinder CVVTL prototype of the engine cylinder head (Figure 2). In the prototype, the timing and lift of the intake valves are adjusted by the CVVTL. For the exhaust valves, only the timing is adjustable. There are one cam cylinder, one phase regulator, and one lift regulator for the intake valves of a cylinder and one cam cylinder and one phase regulator for the exhaust valves of a cylinder.

All intake cam cylinder pistons, which are driven by the intake cam, are laid with a spacing of 90°. All exhaust cam cylinder pistons, which are driven by the exhaust cam, are laid with the same spacing. The intake cam and exhaust cam are mounted on the same camshaft. The angle between the two cams meets the requirement of engine gas distribution. The intake cam cylinders, exhaust cam cylinders, camshaft, intake phase regulators, intake lift regulators, as well as exhaust phase regulators are integrated in the driving assembly.

The intake phase regulators and exhaust phase regulators are controlled by the phase adjusting device, while the intake lift regulators are controlled by the lift adjusting device. The intake and exhaust valve cylinders are integrated in the intake valve cylinder assembly and the exhaust valve cylinder assembly, respectively. The intake valve cylinder assembly and the exhaust valve cylinder assembly are connected with the oil passage assembly via the driving assembly.

The camshaft is driven by the servo motor with the synchronous belt, with a transmission ratio of 1 : 1. The valve motion was measured by the laser displacement sensor. During the experiments, both the phase adjusting device and lift adjusting device were adjusted manually.

## 3. Fluctuation Features and Harms

### 3.1. Fluctuation Features

#### 3.1.1. Different Engine Speeds

Figure 3 shows the system pressure curves at different engine speeds, when neither valve timing nor valve lift is adjusted. When the engine speed was less than 1,716 r/min, the system pressure almost had no fluctuation. When the engine grew continuously beyond that speed, the maximum pressure gradually increased, while the minimum pressure gradually decreased. The faster the engine speed, the more obvious the system pressure fluctuated.

With the rise of engine speed, the crank angle that the system arrives at its minimum pressure became smaller. When the engine moved at 5,150 r/min, the minimum pressure was smaller than the initial pressure, and the second smallest pressure was very close to the initial pressure. It could be predicted that, with further growth of engine speed, the crank angle and the minimum pressure would continue to decrease, and the duration angle and the number of troughs of the system pressure curve would increase.

Once the system pressure fell below the initial pressure, the valve would be out of control. Then, the oil supply subsystem would automatically replenish oil to the system, causing the hydraulic pressure to rise in the system. In this case, the CVVTL would lose its gas distribution capability. Therefore, the CVVTL should work in the engine speed range, which ensures that the system pressure is always greater than the initial pressure. To support the CVVTL operations at a high engine speed, it is necessary to effectively control and mitigate the fluctuation of system pressure.

#### 3.1.2. Different Adjustment Quantities of the Phase Regulator

Figure 4 shows the system pressure curves at three different adjustment quantities of the phase regulator (1 mm, 2 mm, and 3 mm) and the engine speed of 4,006 r/min. As can be seen from the figure, as the adjustment quantity of the phase regulator increased, the maximum system pressure dropped, yet the system pressure fluctuated more significantly. When the adjustment quantity of the phase regulator was greater than 3 mm, the system pressure fell below the initial pressure before the valve opened, and the valve timing could not be effectively adjusted by the CVVTL. Therefore, the adjustment quantity of the phase regulator should be less than 3 mm at 4,006 r/min.

#### 3.1.3. Different Adjustment Quantities of the Lift Regulator

Figure 5 shows the system pressure curves at three different adjustment quantities of the lift regulator (1 mm, 2 mm, and 3 mm) and the engine speed of 4,006 r/min. As can be seen from the figure, as the adjustment quantity of the lift regulator increased, the maximum system pressure dropped and appeared later, the system pressure fluctuated more significantly, and the minimum system pressure declined. If the adjustment quantity of the lift regulator continues to rise, the system pressure would fall below the initial pressure.

#### 3.1.4. Different Pretightening Forces of the Valve Spring

Figure 6 shows the system pressure curves at different pretightening forces of the valve spring at the engine speed of 4,006 r/min. With the growing pretightening force of the valve spring, the system pressure increased, and the trough point of system pressure (i.e., the position of minimum system pressure) moved away from the initial pressure. Hence, the minimum system pressure could be improved by reducing the pretightening force of the valve spring. If that force is too large, more drive energy would get lost, resulting in a greater stress and a more severe wear to hydraulic components.

#### 3.1.5. Different Masses of Valve Components

Figure 7 shows the system pressure curves at different masses of the valve components at the engine speed of 4,006 r/min. With the growing mass of the valve components, the maximum system pressure was on the rise, and the system pressure fluctuated more apparently. Using light valve components can improve the system pressure curve and allow the CVVTL to work at a faster speed.

### 3.2. Fluctuation Harms

The foregoing analysis shows that, when the CVVTL operates faster than the maximum allowable rotational speed, the pressure fluctuation will cause the system pressure to fall below the initial pressure. As the engine speed continues to increase, the system pressure will oscillate more prominently, the valve at the trough point of system pressure will decrease, and the system will eventually enter the negative pressure state. The pressure fluctuation will bring the following harms to the system:

1. Once the system pressure falls below the initial pressure, the valve movement will be out of control, making it hard to adjust the intake air volume of the engine. In this case, the CVVTL cannot meet the engine gas demand.
2. When the system pressure is less than the initial pressure, the oil supply subsystem will automatically replenish the oil to the system, pushing up the system pressure. If too much oil is replenished, the system pressure will exceed the reasonable design range, as the cam returns to the base circle, and the hydraulic force acting on the valve cylinder piston will surpass the valve spring preload. If this occurs, the valve will not be seated, and the engine will not work properly.
3. When the system enters the negative pressure state, the air dissolved in the hydraulic oil will precipitate in the form of bubbles. The ensuing cavitation will compromise the CVVTL. What is worse is that fatigue peeling will take place on the metal parts. Repeated negative pressures will seriously damage the system. In addition, the volume elastic modulus of the oil will nosedive, further weakening the system stiffness. Then, the system vibration will be exacerbated during the high-speed operation.

## 4. Fluctuation Causes

The CVVTL adjusts the valve timing and lift by changing the total volume of the system. Without considering the risk of leakage, the system pressure should be constant and equal to the initial pressure, when the total volume of the system remains constant, that is, the volume change of the cam cylinder equals the total volume change of the valve cylinder, the phase regulator cylinder, and the lift regulator cylinder. If the volume change of the cam cylinder is greater than the said total volume change, the total system volume would shrink, and the oil would be compressed. Then, the system pressure would rise gradually, surpassing the initial pressure. If the volume change of the cam cylinder is smaller than the said total volume change, the total system volume would expand, and the oil volume would grow. Then, the system pressure would fall below the initial pressure. Mathematically, the above change trends can be expressed as

(1) Vc=V+vVp+Vl,p=p0,Vc>V+vVp+Vl,p>p0,Vc<V+vVp+Vl,p<p0,

where *V*_*c*_, *V*_*v*_, *V*_*p*_, and *V*_*l*_ are the volume changes of the cam cylinder, the valve cylinder, the phase regulator cylinder, and the lift regulator cylinder, respectively; *p* is the system pressure; *p*_0_ is the initial pressure.

Figure 8 shows the system pressure curve and volume change curves at the engine speed of 5,500 r/min. Note that Curve 1 is about system pressure; Curve 2 is about the volume change of the cam cylinder; Curve 3 is about the total volume change of the valve cylinder, the phase regulator cylinder, and the lift regulator cylinder; Curve 4 is the cam profile.

In the AB segment, Curve 2 was above Curve 3, and the gap gradually increased. The largest gap between them appeared at point B. This means, in the AB segment, the volume reduction of the cam cylinder is greater than the total volume increment of the valve cylinder, the phase regulator cylinder, and the lift regulator cylinder. Hence, the total system volume gradually decreases, and the oil is compressed. Then, the system pressure would surpass the initial pressure, and gradually approach the maximum pressure, corresponding to the AB segment of Curve 1.

In the BC segment, Curve 2 was still above Curve 3; yet, the gap gradually narrowed. The volume reduction of the cam cylinder equals the said total volume increment at point C. This means, the oil volume compressed in the AB segment gradually expands and returns to the initial volume at point C. Therefore, the system pressure would gradually fall from the maximum pressure at point B to the initial pressure, corresponding to the BC segment of Curve 1.

In the CD segment, Curve 2 was below Curve 3, and the gap gradually widened before shrinking. That is, the volume reduction of the cam cylinder is smaller than the said total volume increment. Hence, the system pressure is less than the initial pressure and would gradually fall and then increase to the initial pressure, corresponding to the CD segment of Curve 1. Then, the system would be replenished by the oil supply subsystem.

In the DE segment, Curve 2 was above Curve 3, namely, the volume reduction of the cam cylinder is greater than the said total volume increment. Note that the gap first gradually increases and then narrows slowly. In this case, the oil would be compressed again and then expanded. Therefore, the system pressure would gradually increase from the initial pressure to the peak, before falling from the peak to the initial pressure. This process corresponds to the DEF segment of Curve 1.

The case of EF segment is the same as that of the CD segment: the system pressure is below the initial pressure and would decrease slowly before a gradual increase, corresponding to the FG segment of Curve 1. Then, the system would be replenished by the oil supply subsystem again.

The case of FG segment is similar to that of the DE segment. Since much oil has been replenished to the hydraulic system, the system pressure would pick up sharply before a gradual decline. In a working cycle, two replenishments happen to the system. Therefore, the system pressure would be larger than the initial pressure when the cam returns to the base circle segment.

The above analysis reveals an important cause of oil pressure fluctuation: the volume reduction of the cam cylinder is not equal to the total volume increment of the valve cylinder, the phase regulator cylinder, and the lift regulator cylinder.

## 5. Countermeasures

With the increase of engine speed, the hydraulic system pressure of the CVVTL will oscillate rather violently, producing a huge pressure shock. Then, the CVVTL operation will be seriously limited, as the engine operates at a fast speed. The system pressure fluctuation can be controlled in two aspects: firstly, prevent excessively large system pressure, or the valve may fly out. Secondly, prevent excessively low system pressure (keep the system not too far below the initial pressure) in the working segment of the cam. Once the system pressure falls below the initial pressure, the oil supply subsystem would start oil replenishment, which affects the next cycle of the engine. If the system enters the negative pressure state, the valve would go out of control, and too much oil would be added to the hydraulic system, making it impossible for the CVVTL to work properly. The system pressure fluctuation must be effectively controlled to ensure the adaptability and reliability of the CVVTL.

### 5.1. Improve the Natural Frequency of the System

The system vibration causes the system oil pressure to vary. This vibration can be reduced by increasing the natural frequency of the system. Thus, this paper suggests curbing the pressure fluctuation of the CVVTL by improving the system natural frequency. The natural frequency of the CVVTL can be expressed as

(2) $$\begin{array}{c} f=\sqrt{\frac{k}{m}}, \end{array}$$

where *f* is the natural frequency of the CVVTL, *k* is the system stiffness, and *m* is the total mass of moving components.

Formula (2) shows that the natural frequency of the CVVTL can be improved by increasing the system stiffness and reducing the total mass of moving components. By the definition of hydraulic system stiffness, the stiffness of the CVVTL can be expressed as

(3) $$\begin{array}{c} k=\frac{F}{\delta }\\ =\frac{\Delta p\cdot A}{\Delta V/A}\\ =\frac{\Delta p}{\Delta V}\cdot A^{2}, \end{array}$$

where *F* is the load of the cam piston, *δ* is the displacement of the cam piston under load, Δ*p* is the increment of system pressure, Δ*V* is the volume change of hydraulic oil, and *A* is the cross-sectional area of the cam piston.

The elastic modulus of the hydraulic oil *E* can be expressed as

(4) $$\begin{array}{c} E=\frac{\Delta p}{\Delta V/V}, \end{array}$$

where *V* is the total volume of the hydraulic oil in the system.

Formula (4) can be rewritten as

(5) $$\begin{array}{c} \frac{\Delta p}{\Delta V}=\frac{E}{V}. \end{array}$$

Substituting formula (5) into formula (3), the system stiffness *k* can be expressed as

(6) $$\begin{array}{c} k=\frac{EA^{2}}{V}. \end{array}$$

Formula (6) shows that, the system stiffness is proportional to the square of the cross-sectional area of the cam piston and the volume elastic modulus of the hydraulic oil in the system while inversely proportional to the total volume of that oil. Therefore, the system stiffness can be improved by expanding the cross-sectional area of the cam piston, reducing the total volume of the hydraulic oil in the system, and using a hydraulic oil with a large volume elastic modulus.

Without considering valve timing adjustment and lift adjustment, the relationship between the valve maximum lift and cam maximum lift can be expressed as

(7) $$\begin{array}{c} \frac{H_{cm}}{H_{vm}}=\sqrt{\frac{A}{A_{V}}}, \end{array}$$

where *H*_*cm*_ is the cam maximum lift, *H*_*vm*_ is the valve maximum lift, and *A*_*v*_ is the cross-sectional area of the valve cylinder piston.

When the valve maximum lift and the cam maximum lift are satisfied, the system stiffness can be improved by using the piston with the largest possible cross-sectional area.

In the specific design, the total volume of the hydraulic oil in the system can be reduced by selecting the size of the oil chamber reasonably, filling the process holes formed in the processing and manufacturing processes, and properly decreasing the length of the oil line.

The volume elastic modulus of the hydraulic oil depends on the temperature and the air content of the oil. It is negatively correlated with the amount of air mixed in it and the temperature level. To reduce the air content, the oil should be directed into the oil tank slowly, such as to prevent the forming of spray or foam in the tank. To control the oil temperature, the hydraulic oil of the CVVTL should be replaced after each working cycle, for the replacement can take away the heat generated in the work of the oil. In this way, it is possible to rationalize the volume elastic modulus of the hydraulic oil.

### 5.2. Parallel a Buffer Accumulator with the System

When the engine runs at a high speed, the system pressure remains high and fluctuates significantly. To ensure the normal operation of the system, it is a must to control the peak pressure and pressure fluctuation of the system. Paralleling a buffer accumulator with the system can both limit the maximum pressure of the system and improve the minimum operating pressure. The structure of the buffer accumulator is shown in Figure 9. The working principle of the buffer accumulator is as follows:

For the buffer accumulator, the pretightening force and stiffness of the spring are selected appropriately based on the needs of the system. The pretightening force must be greater than that of the valve spring so that the valve can open normally. Meanwhile, the stiffness must be smaller than that of the valve spring. When the hydraulic pressure on the buffer accumulator plunger is greater than the pretightening force of the buffer accumulator spring, the piston of the buffer accumulator would move, and the oil would flow into the buffer accumulator rather than into the valve cylinder. In this way, the system pressure would not increase very significantly, putting the maximum pressure under control. When the hydraulic pressure on the buffer accumulator plunger is smaller than the pretightening force of the buffer accumulator spring, the piston of the buffer accumulator would move to the initial position under the action of the spring force. In this case, the oil would flow back into the system from the buffer accumulator. The falling of system pressure would be slowed down, making the system pressure more stable.

Figure 10 shows the system pressure curves and valve lift curves at the engine speed of 5,500 r/min. Note that Curve 1 is the valve lift curve of the CVVTL without the parallelization of the buffer accumulator; Curve 2 is the valve lift curve of the CVVTL paralleled with a buffer accumulator; Curve 3 is the system pressure curve of the CVVTL without the parallelization of the buffer accumulator; Curve 4 is the system pressure curve of the CVVTL paralleled with a buffer accumulator.

As shown in Figure 10, Curve 3 had a greater maximum hydraulic pressure, fewer fluctuation numbers, and a larger amplitude than Curve 4. In Curve 3, two troughs were less than the initial pressure, and the valve lift peaked at 11.25. In Curve 4, the maximum valve lift was 10.28, smaller than that in Curve 3. These results demonstrate that the CVVTL can effectively control the pressure fluctuation and the maximum valve lift and improve the maximum allowable working speed of the CVVTL after the system is paralleled with a buffer accumulator.

### 5.3. Choose Reasonable Design Parameters

The design parameters directly bear on the CVVTL performance, including but not limited to the mass of valve components, the pretightening force and stiffness of the valve spring, the parameters of the lift regulator, the parameters of the phase regulator, and the length and diameter of the hydraulic pipe. Choosing the reasonable design parameters would significantly improve the system pressure fluctuation.

### 5.4. Design Reasonable Cam Profile

Cam, the power source of the hydraulic system, drives the system by the cam cylinder piston. The motion rule of the cam profile affects the fluctuation of the system pressure and the movement law of the valve. Therefore, the system pressure fluctuation can be improved by designing the cam profile more rationally. Possible design measures include selecting a cam profile with a continuous acceleration curve (e.g., a high-power cam profile), reducing the maximum acceleration of the cam profile, and widening the positive speed cam profile. In considering the system working characteristics of the system, the design method of cam profile should not only meet the basic requirements of inflation efficiency, contact stress, and smooth operation, etc. but it can also meet the special design requirements of valve adjustment matching and oil compression compensation.

According to the above analysis results, the mechanism parameters of the system are optimized. The recaptured system pressure fluctuation test curves are shown in Figure 11. Compared with Figure 3, the fluctuation range of oil pressure is significantly reduced. When the engine speed reaches 5500 r/min, the fluctuation range is 1.3∼8.9 MPa, both higher than the initial oil pressure of the system.

## 6. Conclusions

In the proposed CVVTL, the system pressure fluctuates more violently with the increase of the engine speed. The minimum (trough value) of system pressure equals the initial pressure when the engine speed reaches the maximum allowable value. Further increase in engine speed would throw the system into the negative pressure state. Then, the CVVTL will lose its distribution capability. The system pressure fluctuation is affected by multiple factors such as the adjustment quantity of the phase regulator, the adjustment quantity of the lift regulator, the pretightening force and stiffness of the valve spring, and the mass of the valve components. It limits the maximum operating speed of the CVVTL.

The fluctuation of the oil pressure is primarily caused by the fact that the volume reduction of the cam cylinder is not equal to the total volume increment of the valve cylinder, the phase regulator cylinder, and the lift regulator cylinder.

The fluctuation of system pressure can be effectively controlled by improving the natural frequency of the system, paralleling a buffer accumulator with the system, choosing reasonable design parameters, and designing reasonable cam profile.

The fluctuation range of oil pressure is significantly reduced to 1.3∼8.9 MPa, which increases the applicable range of CVVTL to 5,500 r/min.

## Figures and Tables

**Figure 1:** System structure.

**Figure 2:** CVVTL prototype.

**Figure 3:** System pressure curves at different engine speeds.

**Figure 4:** System pressure curves of different adjustment quantities of the phase regulator.

**Figure 5:** System pressure curves of different adjustment quantities of the lift regulator.

**Figure 6:** System pressure curves at different pretightening forces of the valve spring.

**Figure 7:** System pressure curves at different masses valve component.

**Figure 8:** System pressure curve and volume change curves at the engine speed of 5,500 r/min.

**Figure 9:** Structure of the buffer accumulator.

**Figure 10:** System pressure curves and valve lift curves at the engine speed of 5,500 r/min.

**Figure 11:** System pressure curves at different engine speeds.

**Table 1:** Optimal gas distribution parameters at different engine speeds.

Engine speed (r/min)	IVO (deg)	IVC (deg)	Valve lift (mm)
1500	82	302	7.24
2500	83	310	7.71
3500	79	318	7.81
4500	73	335	8.54
5500	77	348	8.76

## Data Availability

No data were used to support this study.
